# SR-DSFF and FENet-ReID: A Two-Stage Approach for Cross Resolution Person Re-Identification

**DOI:** 10.1155/2022/4398727

**Published:** 2022-07-05

**Authors:** Zongzong Wu, Xiangchun Yu, Donglin Zhu, Qingwei Pang, Shitao Shen, Teng Ma, Jian Zheng

**Affiliations:** ^1^Jiangxi University of Science and Technology, Ganzhou, Jiangxi 341000, China; ^2^Xi'an Zhongtie Rail Transit Co., Ltd., Xian, Shaanxi 710000, China

## Abstract

In real-life scenarios, the accuracy of person re-identification (Re-ID) is subject to the limitation of camera hardware conditions and the change of image resolution caused by factors such as camera focusing errors. People call this problem cross-resolution person Re-ID. In this paper, we improve the recognition accuracy of cross-resolution person Re-ID by enhancing the image enhancement network and feature extraction network. Specifically, we treat cross-resolution person Re-ID as a two-stage task: the first stage is the image enhancement stage, and we propose a Super-Resolution Dual-Stream Feature Fusion sub-network, named SR-DSFF, which contains SR module and DSFF module. The SR-DSFF utilizes the SR module recovers the resolution of the low-resolution (LR) images and then obtains the feature maps of the LR images and super-resolution (SR) images, respectively, through the dual-stream feature fusion with learned weights extracts and fuses feature maps from LR and SR images in the DSFF module. At the end of SR-DSFF, we set a transposed convolution to visualize the feature maps into images. The second stage is the feature acquisition stage. We design a global-local feature extraction network guided by human pose estimation, named FENet-ReID. The FENet-ReID obtains the final features through multistage feature extraction and multiscale feature fusion for the Re-ID task. The two stages complement each other, making the final pedestrian feature representation has the advantage of accurate identification compared with other methods. Experimental results show that our method improves significantly compared with some state-of-the-art methods.

## 1. Introduction 

The purpose of person Re-ID is to match the target person of interest across the images under multiple cameras. Due to its wide range of applications, such as intelligent surveillance, person tracking, and criminal case forensics, it has been widely used in computer vision in recent years. With the development of deep learning, many deep feature extraction networks have been designed for person Re-ID to improve the matching accuracy. However, in practical applications, person Re-ID still presents enormous challenges due to factors such as different low-resolution images [1], illumination changes [2], occlusions [3], and weather changes [4].

Some deep learning based person Re-ID methods [5, 6] perform well on the premise of ensuring that the resolutions of gallery images and query images are consistent and high-resolution (HR). However, this premise is usually not guaranteed because the resolution of the query images is usually low, but the gallery images are all filtered HR images, which resulted in a mismatch between the resolution of the query images and gallery images. At this time, traditional person Re-ID methods cannot extract discriminative person features for target matching, so more and more people begin to focus on cross-resolution person Re-ID [7–12]. Cross-resolution person Re-ID works aim to address the problem of resolution mismatch between query images and gallery images.

Cross-resolution person Re-ID was first proposed by Li et al. [13] in 2015, which opened a precedent for cross-resolution person Re-ID research. Subsequent research on cross-resolution person Re-ID can be divided into two stages in time. In some early works, dictionary learning or metric learning are used to learn pedestrians between images of different resolutions. The common feature representations are as shown in work [7–10]. However, the feature maps extracted by these methods based on LR images are unreliable, so the early cross-resolution person Re-ID matching accuracy is not satisfactory. Subsequently, with the proposal of some SR models [14–17], some researchers began to apply SR models to cross-resolution person Re-ID, which is the development of cross-resolution person Re-ID second stage. Jiao et al. [12] were the first to use SRCNN [18] to recover the resolution of LR images and proposed a method to train the SR sub-network and the Re-ID sub-network jointly. Since then, more and more works have begun introducing SR modules into cross-resolution person Re-ID, which further improves the matching accuracy of cross-resolution person Re-ID. For example, MMSR [19] designed a mixed-space super-resolution model to recover the resolution of LR images with variable resolution. Recently, many new methods represented by PRI [11] have improved the detection accuracy of cross-resolution person Re-ID to a new level. However, there are still some gaps in practical application.

Through the study of numerous cross-resolution person Re-ID methods in recent years, we found some of their disadvantages. Most of the current research ideas are to use the SR module to recover the query images resolution to the high-resolution displayed by the gallery images. The use of the SR modules significantly improves the matching accuracy of cross-resolution person Re-ID, but in fact, we found through experiments that the SR images generated after the SR modules will inevitably lose some original details [20]. We believe that this will bring hidden dangers to subsequent Re-ID tasks. Although Zhuang et al. [21] proposed CAD-NET to jointly learn the feature maps of the SR images and the LR images to alleviate the loss of feature details; however, there are still significant problems in directly fusing feature maps from images of different resolutions. Furthermore, most researchers use deep neural networks to capture low-level details by extracting local features [22] of images, which are likely to bring semantic ambiguity. For example, a man with a woman's suitcase is mistaken for a woman. Therefore, we believe that it is necessary to devise better methods in reducing the loss of original details brought by the SR module and extracting image feature extraction.

In this paper, we propose a person Re-ID method that jointly optimizes the feature details of person images and the extraction of features. Specifically, we propose a deep network consisting of the SR-DSFF sub-network and the FENet-ReID sub-network. Firstly, the SR-DSFF uses a dynamic upscale module to learn the weights in the convolution kernel; these weights are then used to generate SR images. Different from other methods that utilize SR models, we treat SR-DSFF as an image enhancement model rather than a single SR model. Therefore, we added the DSFF module after the SR module. The DSFF module clearly distinguishes high- and low-resolution inputs during feature learning, so that the feature information of different resolution images complement each other to ensure its robustness to resolution variance. Subsequently, the global-local feature extraction network (FENet-ReID) extracts person representations for person Re-ID. The FENet-ReID consists of two convolution stages (FE-C1 and FE-C2) and three feature fusion units. The two convolution stages consist of four CNN sub-networks, and each feature fusion unit sequentially fuses two equal-sized feature maps to obtain a more discriminative final feature representation of a person. The main contributions of this paper are as follows:

- We propose an image enhancement sub-network named SR-DSFF. Unlike other methods, we do not rely on a single SR module to recover image resolution. Instead, the DSFF module is added after the SR module to reduce the loss of image details.
- We propose a feature extraction network based on human pose estimation named FENet-ReID, using the final features from multistage feature extraction and multiscale feature fusion to perform cross-resolution person Re-ID.
- We have done a lot of experiments on three cross-resolution person Re-ID datasets, all of which have reached the industry-leading level. Compared with other state-of-the-art methods, our proposed method achieves 2.7%, 5.4%, and 3.7% improvement on Rank-1 on MLR-Market1501, MLR-CUHK03, and CAVIAR datasets, respectively.

The rest of this article is organized as follows: Section 2 introduces the related work and Section 3 mainly introduces the proposed method.  Section 4 evaluates the model's performance through extensive experiments and concludes with a conclusion in Section 5.

## 2. Related Work

### 2.1. Person Re-ID

Person Re-ID has been studied by academia for many years since 2005. Still, it was not until 2014 that deep learning began to be applied to person Re-ID, that person Re-ID achieved a huge breakthrough. Many current methods [23–27] have achieved outstanding results in closed-world [28], and even some state-of-the-art methods have achieved accuracy close to or surpassing the human level. For example, Zheng et al. [29] proposed a method that combines the similarity of intraclass data in high-dimensional space and the difference between classes and achieves complementary effects by fusing the two loss functions. And Chen et al. [30] proposed a method on transfer learning in unsupervised situations, for the two models with the same network to fill the unlabeled part of each other and it can be further replaced by two different networks. As a result, traditional person Re-ID has entered a bottleneck period and many methods have been developed to deal with various challenges, such as pedestrians with different poses, different styles of cameras, and occlusion. For example, Wei et al. [31] proposed a GLAD that exploits both local and global features of the human body to generate a representation with strong discriminativeness to handle significant variations in human poses. Liu et al. [32] proposed a method for uniform style, that is, to deal with the style changes caused by different cameras by generating images with a unified camera style through Unity GAN. Qian et al. [33] proposed a generative adversarial network (PNGAN) specially designed for pose normalization in Re-ID. Some methods [34–36] use human pose information to reduce background noise to solve the problem of occlusion. However, the above methods usually assume that the resolutions of query images and gallery images are similar and high enough, which will bring significant problems to applying these methods in open-world [28].

### 2.2. Cross-Resolution Person Re-ID

In order to solve the problem that the resolution span is too large, many methods have also been proposed in recent years. Traditional methods [37, 38] process images employing metric learning or dictionary learning, but the details of LR images are not obvious, so the performance of these methods is limited. With the development of super-resolution technology, some SR-based cross-resolution person Re-ID methods have been proposed in later studies. SR-based cross-resolution person Re-ID usually relies on SR modules to recover the resolution of LR images. Since Ledig et al. [16] first proposed SRGAN, SR modules have been widely used in the resolution recovery stage of cross-resolution person Re-ID. And Jiao et al. [12] jointly trained SRCNN and Re-ID networks for the first time. Mao et al. [39] proposed a Foreground-Focus Super-Resolution (FFSR) module and Resolution-Invariant Feature Extractor (RIFE). Unlike other SR-based methods, FFSR combines Re-ID loss and foreground attention loss during training and suppresses irrelevant background while restoring pedestrian image resolution. Some other SR models are also widely used in cross-resolution person Re-ID, such as Meta-SR [17] and VDSR [40].

### 2.3. Feature Representation Learning in Person Re-ID

In the field of person Re-ID, most deep learning based works [41–43] are used to extract feature maps from the entire pedestrian images, so simply extracting global features is likely to lose key information about pedestrians. Subsequent works [44–46] tried to horizontally divide pedestrian images into several fixed-length blocks to extract more detailed local features. The experimental results show that the matching accuracy of person Re-ID after adding local features is much better than those methods that use global features. However, dividing the pedestrian image into fixed-length blocks to extract local features is not sensitive to the change of the pedestrian's posture. The pedestrians captured by the surveillance cameras often have posture changes. Therefore, it is necessary to design a better feature extractor for pedestrian pose changes.

### 2.4. Discussion

Cross-resolution person Re-ID is only a branch of the field of person Re-ID. There are still many issues to be resolved. For example, to make the person Re-ID technology applicable on a large scale, we need to design a lighter network while ensuring the accuracy so that the hardware device can accept it. In addition, in the research of person Re-ID, I found that some techniques can also be applied to building retrieval [47] or drone-based geo-localization [48] etc.

At present, most SR-based cross-resolution person Re-ID methods focus on the reconstruction of SR images so the reconstructed SR images can be closer to the original HR images. However, these methods ignore the loss of image detail in the reconstruction process and the distribution difference between high- and low-resolution image features. Different from current methods, our network learns and fuses features from LR and HR images through dual-streams of attention-weighted feature extraction while recovering the image resolution. Compared with the way current methods deal with LR images, our method preserves richer image feature details.

## 3. Proposed Methods

Our network structure diagram is shown in Figure 1. This section introduces the SR-DSFF and FENet-ReID, respectively.

### 3.1. SR-DSFF

As the first stage of cross-resolution person Re-ID, we first consider restoring the resolution of the query images. For open-world, we often face the problem that the resolution span of query images is too large, so we cannot predict a suitable scale factor to handle query images of arbitrary resolutions. For open-world needs and improving cross-resolution person Re-ID methods, it is crucial to design a method that can handle query images at arbitrary resolutions. Inspired by some work [49], we employ a dynamic Meta-Upscale module to learn the weights in the convolution kernels, which are then used to generate SR images. Our SR module is different from some existing SR models such as FSRCNN [14], SRDenseNet [15], and SRGAN [16]. Inspired by meta-learning [50], we divide the SR module into two modules, the feature learning module and the Meta-Upscale module [17]. We choose RDN [51] as the feature learning module, and it is worth noting that we replace the ordinary upscale module with an improved Meta-Upscale module.

SR-DSFF takes a set of LR images *I*_*L*_^*n*^={*I*_*L*_^1^, *I*_*L*_^2^, *I*_*L*_^3^,…, *I*_*L*_^*N*^} as input. In the training phase, we obtain images *I*_*L*_^*n*^ from a set of original HR images *I*_*H*_^*n*^={*I*_*H*_^1^, *I*_*H*_^2^, *I*_*H*_^3^,…, *I*_*H*_^*N*^} by down-sampling. In the SR module, our goal is to predict the SR images *I*_*S*_^*n*^={*I*_*S*_^1^, *I*_*S*_^2^, *I*_*S*_^3^,…, *I*_*S*_^*N*^} from images *I*_*L*_^*n*^. Assuming that the scale factor of each pixel (*i*_1_, *j*_1_) of the images *I*_*L*_^*n*^ is *s* during the enlargement process, in the prediction stage, the features *F*_*IL*_^*n*^ of the images *I*_*L*_^*n*^ is extracted by the feature learning module in the SR module, The features of the images *I*_*L*_^*n*^ on its pixel (*i*_1_, *j*_1_) and the corresponding filter weights determine each pixel (*i*, *j*) in the generated images *I*_*S*_^*n*^.

For each pixel (*i*, *j*) in the images *I*_*S*_^*n*^, it is determined by the feature of the images *I*_*L*_^*n*^ on its pixel (*i*_1_, *j*_1_) and the corresponding filter weights. So we can think of the Meta-Upscale module as a mapping function from *F*_*IL*_ to *I*_*S*_^*n*^. The mapping function is as follows:

(1) $$\begin{array}{c} I_{S}^{n}\left(i,j\right)=f\left(F_{IL}^{n}\left(i_{1},j_{1}\right),\;w\left(i,j\right)\right), \end{array}$$

where *I*_*S*_^*n*^(*i*, *j*) is the pixel value of the images *I*_*S*_^*n*^ at (*i*, *j*), *f*(  *·*  ) represents the feature mapping function for calculating pixel values, and *w*(*i*, *j*) is the weight prediction module of the pixel point (*i*, *j*) (corresponding to equation (3)).

For each pixel (*i*, *j*) in the images *I*_*S*_^*n*^, we consider the pixel (*i*, *j*) to be determined by the features of (*i*_1_, *j*_1_) on the LR images. We map these two pixels through a projection transformation function *T*:

(2) $$\begin{array}{c} \left(i_{1},j_{1}\right)=T\left(i,j\right)=\left(\frac{i}{s},\frac{j}{s}\right). \end{array}$$

Specifically, we can think of the resolution recovery process as a variable fractional stride mechanism that enables convolution to use an arbitrary scale factor *s* (not limited to integer multiples of scale factors) to upscale feature maps. For example, when the scale factor *s*=2, one pixel (*i*_1_, *j*_1_) determines two pixels on the images *I*_*S*_^*n*^. If the scale factor is a non-integer, taking *s*=1.5 as an example, some pixels determine two pixels, and some pixels determine one pixel. All in all, each pixel (*i*, *j*) on the images *I*_*S*_^*n*^ can find a most relevant pixel (*i*_1_, *j*_1_) on the images *I*_*L*_^*n*^.

After determining the positional relationship between the images *I*_*L*_^*n*^ and the images *I*_*S*_^*n*^, it is also necessary to learn the weights and offset between the two. Different from the traditional upscale module, our Meta-Upscale module predicts the corresponding number of filter weights for any scale factors employing two fully connected layers. In order to train multiple scale factors simultaneously, it is better to add the scale factors to *v*_*ij*_ to distinguish the weights of different scale factors. We can express the weight prediction and *v*_*ij*_ as follows:

(3) $$\begin{array}{c} W\left(i,j\right)=\varphi \left(v_{ij};\theta \right), \end{array}$$

(4) $$\begin{array}{c} v_{ij}=\left(\frac{i}{s}-\frac{i}{s},\frac{j}{s}-\frac{j}{s}\right), \end{array}$$

where *W*(*i*, *j*) is the convolution kernel weight corresponding to the pixel (*i*, *j*) on the images *I*_*S*_^*n*^, *v*_*ij*_ is the vector associated with (*i*, *j*), *φ* is the weight prediction network, and *θ* is the weight of the weight prediction network. Then obtain the pixel value of the pixel (*i*_1_, *j*_1_). Its feature mapping function is expressed as follows:

(5) $$\begin{array}{c} \Phi \left(F_{IL}\left(i_{1},j_{1}\right),W\left(i,j\right)\right)=\;F_{IL}\left(i_{1},j_{1}\right)W\left(i,j\right). \end{array}$$

Finally, in order to ensure that the images *I*_*S*_^*n*^ have high-resolution, we define a SR loss ℒ_rec_ between the SR images and its original HR images, and the SR loss ℒ_rec_ is expressed as follows:

(6) $$\begin{array}{c} {ℒ}_{\text{rec}}=E\left[\left\|I_{S}^{n}-I_{H1}^{n}\right\|\right], \end{array}$$

where *I*_*H*_^*n*^ and *I*_*S*_^*n*^ represent original HR images and SR images, respectively. As shown in Figure 2, the effect of the SR module on the resolution recovery of LR images is pronounced.

It is worth noting that although we use the SR loss ℒ_rec_ to make the images *I*_*S*_^*n*^ to reduce the loss of pedestrian features during the resolution recovery process. However, in the process of resolution recovery, the loss of features is still inevitable. In addition, the visual cues contained between different resolution images are different, so it is not reliable to rely on the SR images for the Re-ID task. To sum up, we added a DSFF module after the SR module to learn the features in different resolution images *I*_*L*_^*n*^ and *I*_*S*_^*n*^ and fuse the learned feature maps. Since SR images and LR images contain other visual cues, different feature extractors should be used to extract image feature maps of different resolution images.

The DSFF module consists of two feature extraction branches. We denote these two branches named FES^*L*^ and FES^*S*^, respectively. In each branch, we take ResNet101 [52] as the backbone, and ResNet101 is modified to be a Feature Extraction Block named FEB to extract the feature maps of the input images by duplicating its convolutional layers as FES^*L*^ and FES^*S*^. And we introduce spatial attention and channel attention in FES^*L*^ and FES^*S*^. As shown in Figure 1, there is always a feature extraction branch in FEB corresponding to the images *I*_*L*_^*n*^ and images *I*_*S*_^*n*^, respectively. Among them, FES^*L*^ and FES^*S*^ have the same structure. However, the training purposes of the two branches are different. For example, for the SR images, we choose a more appropriate FES^*S*^ for feature extraction, so the *m*^*S*^ is fused with larger weights. As shown in Figure 3, in the spatial attention, we utilize softmax to transform the learned feature vectors into weight *ω*^*L*1^ or *ω*^*S*1^, in the channel attention, we use one global average pooling (GAP) layer and two fully connected (FC) layers to predict *ω*^*L*2^ or *ω*^*S*2^, and the feature maps *m*^*L*^ and *m*^*S*^ obtained by each branch can be expressed as follows:

(7) $$\begin{array}{c} m^{L}=\omega^{\text{L}1}\times m^{L1}+\omega^{\text{L}2}\times m^{L2}, \end{array}$$

(8) $$\begin{array}{c} m^{S}=\omega^{\text{S}1}\times m^{S1}+\omega^{\text{S}2}\times m^{S2}, \end{array}$$

where *m*^*L*^ and *m*^*S*^ represent feature maps obtained by FES^*L*^ and FES^*S*^, respectively. *m*^*L*1^ and *m*^*L*2^ represent the feature maps obtained by FES^*L*^ through spatial attention and channel attention, respectively. *m*^*S*1^ and *m*^*S*2^ represent the feature maps obtained by FES^*L*^ through spatial attention and channel attention, respectively. The resolution of the input images determines the size of *ω*^*L*^ and *ω*^*S*^. For LR images, *ω*^*L*^ will be larger than *ω*^*S*^, and vice versa. In order to learn *ω*^*L*^ and *ω*^*S*^, we introduce resolution weighting loss ℒ^*R*^. According to the training images *I*_*L*_^*n*^ and *I*_*S*_^*n*^ can be expressed as follows:

(9) $$\begin{array}{c} {ℒ}^{R}\left(I_{r}^{n}\right)={\left\|\omega^{L}-\left(1-r\right)\right\|}_{2}^{2}+{\left\|\omega^{S}-r\right\|}_{2}^{2}, \end{array}$$

where *ω*^*L*^=(*ω*^*L*1^, *ω*^*L*2^), *ω*^*S*^=(*ω*^*S*1^, *ω*^*S*2^), *I*_*r*_^*n*^ represents *I*_*L*_^*n*^ or *I*_*S*_^*n*^, and *r* represents the resolution of *I*_*r*_^*n*^. Finally, we denote the output feature *m* as follows:

(10) $$\begin{array}{c} m\;=\;m^{L}+\;m^{S}. \end{array}$$

Finally, the feature **m** is put into the last transposed convolutional layer of the SR-DSFF to get the final image with richer semantic information.

### 3.2. FENet-ReID

After obtaining the final images, our ultimate goal is to obtain a discriminative pedestrian feature representation for the Re-ID task. To get this feature map as shown in Figure 1, we extract global and local features from the final images and fuse them.

We utilize human pose estimation [53]. Unlike Spindie Net [54], we only select four key points on pedestrians to make our model robust to a wider variety of pedestrian poses and camera views. Based on these four key points, we get three key regions of pedestrians: the head, upper body, and lower body.

Our FENet-ReID process consists of two modules, the Feature Extraction Module (FEM) and the Feature Fusion Module (FFM). The FEM and FFM are introduced separately below.

#### 3.2.1. FEM

We design a Convolutional Neural Networks (CNNs) consisting of four sub-networks in FEM. As shown in Figure 4, the FEM consists of two convolution stages (FE-C1 and FE-C2). Using the FEM, we obtain four 256-dimensional feature vectors from the pedestrian image global and three key regions. In FE-C1, there are three convolutional layers and one Inception module [55] in each CNN. First, convolve the input image to obtain a feature map with a spatial size of 24 × 24. At the same time, the same operation is performed on the three key regions of pedestrian and a ROI Pooling operation is performed to keep the feature maps obtained by FE-C1 of equal size. In FE-C2, the four feature maps obtained in the previous stage are input, and the spatial size is reduced to 12 × 12 through an initial module first, then we use a global pooling layer and a fully connected layer to convert into 256-dimensional feature vectors, that is, the output of FE-C2 is four 256-dimensional feature vectors, which correspond to the global image and three human key regions images, respectively.

#### 3.2.2. FFM

To make the final feature representation of pedestrians more discriminative, next we fuse together the four 256-dimensional feature vectors obtained earlier to generate a compact 256-dimensional feature vector. We adopt a feature fusion unit to fuse two feature vectors of equal size. Specifically, as shown in the right part of Figure 4, we use three such feature fusion units, where two primary operations are performed in each feature fusion unit: (1) Use the element-wise maximization operation to delete the features of the smaller value, and only keep the features of the maximum value. (2) An inner product layer is used for feature transformation, and its output can be used for subsequent feature fusion units. The three feature fusion units from left to right sequentially fuse the pedestrian's lower body and upper body into the main body, fuse the main body and head into the whole body, and finally fuse the whole body and feature vector of the full image into the final 256-dimensional feature *F*. Finally, we use a fully connected layer on the feature *F* to predict the ID labels of pedestrians. It can be expressed as person Re-ID loss by a cross-entropy loss ℒ^*X*^, and the expression is as follows:

(11) $$\begin{array}{c} {ℒ}^{X}\left(I_{n}\right)=\text{CrossEntropy}\left(FC\left(F_{n}\right),P_{n}\right), \end{array}$$

where *I*_*n*_ represents the final images obtained by transposed convolution in SR-DSFF and *P*_*n*_ represents the person ID labels of the training images *I*_*n*_.

Through a training set *ℤ*={(*I*_*H*_^*n*^, *I*_*r*_^*n*^, *I*_*n*_, *P*_*n*_)}, *n*=1,…, *N*, where *I*_*H*_^*n*^ represents the original HR images, *I*_*r*_^*n*^ represents *I*_*L*_^*n*^ or *I*_*S*_^*n*^, and *P*_*n*_ is the person ID label. The total loss ℒ_TOTAL_ of the DSFF module and FENet-ReID can be expressed as follows:

(12) $$\begin{array}{c} {ℒ}_{\text{TOTAL}}={ℒ}^{X}\left(I_{n}\right)+\alpha \sum_{t=1:4}{ℒ}_{t}^{R}\left(I_{r}^{n}\right), \end{array}$$

where *I*_*r*_^*n*^ means *I*_*L*_^*n*^ or *I*_*S*_^*n*^ input into FES^*L*^ or FES^*S*^.

## 4. Experiment

### 4.1. Dataset

We evaluate our method on three datasets, all of which are most commonly used for person Re-ID.

MLR-Market1501 [56]: Market1501 dataset was captured by six cameras, five of which were high-resolution cameras, and one was low-resolution. Market1501 contains 1501 different pedestrian categories with 32668 detected pedestrian bounding boxes. Among them, pedestrians of each category are captured by at least two cameras. We follow SING [12] that the images captured by one of the cameras are processed at the same down-sampling rate and the resolutions of the images captured by the other cameras remain unchanged to create the MLR-Market1501. Based on the person ID labels, we split the dataset into a training set containing 751 pedestrians and a test set containing 750 pedestrians.

CAVIAR [57] was collected in the real world, including 1220 images of 72 pedestrians captured by two cameras. According to [12], we discarded 22 identities of pedestrian images so that only HR images are included in the dataset. We randomly split the dataset into two training and test sets containing 25 pedestrian identities.

MLR-CUHK03: CUHK03 [58] is the first large-scale person Re-ID dataset, and its colossal data volume is enough to support it for deep learning. The dataset contains 632 different pedestrian categories and is photographed by five pairs of cameras. Also, according to [12], we randomly down-sample the images captured by one of the cameras of each team with the down-sampling rate of *r* ∈ {2,  3,  4} to create the MLR-CUHK03 dataset. We use the same number of pedestrian identities (316/316) as training/testing sets.

### 4.2. Implementation Details

Our model training is divided into two steps: (1) Firstly train the SR module separately and (2) then jointly train the DSFF and FENet-ReID.

In the SR module, the widely used loss function is *L*2 loss, but according to work [59], we use *L*1 loss to make the network better convergence. In the network training, in order to construct the LR image training set, we conduct the down-sampling operation on the images in several data sets and then adjust the image obtained by down-sampling to the same size as the original HR images. It is worth noting that we use a unified down-sampling factor *r* = 4 to down-sample original HR images. For each batch, we randomly selected 16 LR images of 96*∗*96 size as training images. We use Adam as the optimizer. During the training process, the training scale factor of the SR module varies from 1 to 4 with a step of 0.1, and these scale factors are uniformly distributed. Initialize the learning rate of all layers to 10^−4^ and perform 10^6^ update iterations.

DSFF and FENet-ReID are trained by Stochastic Gradient Descent (SGD), and the training is done in two steps: (1) Use ℒ^*R*^ to initialize on the target dataset and adjust the DSFF module. (2) Under the guidance of the loss function in equation (12), the DSFF and FEFF are jointly trained. According to the experiment, we fix the hyper parameter in equation (12) as *α*=1, and each step has 60 epochs, the batch size is set to 32. The initial learning rate is set to 10^−2^ in the first 30 epochs, and 10^−3^ after 30 epochs. The final 256-dimensional feature is used for Re-ID with Euclidean distance.

Our network is trained on Pytorch, and all experiments are implemented with NVIDIA RTX3080Ti GPU, Intel i9 CPU, and 64 GB memory.

### 4.3. Comparison with State-of-the-Art

Tables 1–3 shows the results of our method on three datasets, as well as the comparison with other state-of-the-art methods in the last three years. The methods we choose cover two broad categories: (1) Traditional person re-id methods: SpreID [60], CamStyle [61], LA-Transformer [64]; (2) Advanced methods for cross-resolution person Re-ID (other methods in Tables 1–3). It can be seen from the comparison results that the performance of our method has improved significantly.

On the MLR-Market1501 dataset, the Rank-1 accuracy of our method improves by 2.7% over the current state-of-the-art methods. On the MLR-CUHK03 dataset, compared with other methods, the accuracy is improved by 5.4% relative to second place in Rank-1. On the CAVIAR dataset, our Rank-1 accuracy is also 3.9% better than the current state-of-the-art. It can be seen that SR-DSFF and FENet-ReID outperform the vast majority of existing methods compared with existing cross-resolution person re-id methods. Only on dataset MLR-Market1501 and MLR-CUHK03, our method is on par with LA-Transformer [64] and PRI [11] in Rank-5 accuracy comparison.

### 4.4. Ablation Study

#### 4.4.1. Validity of DSFF and FENet-ReID

To verify the effectiveness of our SR-DSFF and FENet-ReID, as shown in Table 4, we fixed the DSFF as ResNet101 and compared it with other different SR models as shown in Table 5. It is worth noting that we use the entire SR-DSFF as an image enhancement model, because the purpose of our SR-DSFF is to obtain images that are more suitable for person Re-ID. Experiments are performed on the dataset MLR-Market1501.

In Table 4, we fix the DSFF as bilinear interpolation and compare it with three feature extractors, namely, (1) ResNet101 baseline, (2) two ResNet101 with the same weights, and (3) two ResNet101, and dual-stream feature fusion with the learned weights learned by equation (9). From Table 4, we can see that using two ResNet101 improves the model significantly. After further assigning weights to the two ResNet101, the effect also enhances. Finally, our SR-DSFF shows the best results with dual-stream feature fusion and learned weights. The accuracy of Rank-1 is enhanced by 12.3% compared to the baseline.

In Table 5, we discuss the effect of different loss functions on the recognition accuracy of the network. In addition to the loss function we adopted, we also selected three other commonly used loss functions (Circle loss, Triplet loss, and Sphere loss). In the experimental design, we use the exact same SR-DSFF and FENet-ReID and only replace the person Re-ID loss (equation (11)) with other loss functions during network training. Experimental results show that our loss function has the best performance on FENet-ReID guided by human pose estimation.

In Table 6, our method and variants of our method (trained with/without and “weighting loss”) are compared with other SR-based person Re-ID methods. It can be seen from Table 5 that adding weighting loss during training greatly improves the accuracy of Re-ID. At the same time, our method significantly improves the performance of other SR-based cross-resolution person Re-ID methods.

## 5. Conclusion

In this paper, a deep network composed of SR-DSFF and FENet-ReID is proposed to solve the cross-resolution person Re-ID problem. That is a new idea for solving cross-resolution person Re-ID problem, that is, in SR-DSFF, the dynamic Meta-Upscale module is used to recover the LR images to SR images in the SR module, and through the dual-weighted feature extraction stream in the DSFF, the fusion feature maps with more effective pedestrian information are obtained, and the final images is recovered through the transposed convolution. Then, the FENet-ReID is used to segment the three key regions of the person based on the human posture estimation, and the feature extraction is carried out combined with the full images and key region images for person Re-ID. We conducted extensive experiments on three datasets to verify the effectiveness of the proposed method.

## Figures and Tables

**Figure 1:** The network consists of SR-DSFF sub-network and FENet-ReID. The query images first enter the SR-DSFF, and the SR images are output through the feature extractor and the upscale module in the SR module. Then, the feature maps of the query images and the SR images are jointly learned and fused through the DSFF module, and the final images are output into FENet-ReID through transposed convolution. FENet-ReID extracts the global and local features of the images that are obtained in the SR-DSFF and fuses them to obtain the final feature maps. Finally, a fully connected (FC) layer is used on the final feature maps to predict the ID labels of pedestrians. Our network is divided into two training stages: (1) Update the SR module with the SR loss ℒ_rec_ (equation (6)); and (2) jointly train the DSFF and the FENet-ReID with the total loss ℒ_TOTAL_ (equation (12)). These two stages are represented by yellow and black arrows on the figure, respectively.

**Figure 2:** Shows the performance of our SR module on the dataset Market1501. The effect is evident by comparing it with LR images.

**Figure 3:** We add spatial attention and channel attention to the last ResNet101 Block. The lower right corner of the figure takes the branch FES^*L*^ as an example to give a detailed attention diagram, which is in FES^*S*^ has the same structure.

**Figure 4:** Flowchart of FENet-ReID. The full image and three human key regions images are extracted by FE-C1 and FE-C2, respectively, and the obtained 256-dimensional features are fused by three fusion units in FFM.

**Table 1:** The proposed method is compared with the current state-of-the-art methods on the dataset MLR-Market1501.

Methods	MLR-Market1501		
	Rank-1	Rank-5	Rank-10
SING [12]	74.4	87.8	91.6
SPreID [60]	77.4	89	93.9
CamStyle [61]	74.5	88.5	92.2
CAD-net [62]	83.7	92.7	95.8
FFSR + RIFE [39]	66.9	84.7	-
CRGAN [63]	83.7	92.7	95.8
INTACT [22]	**88.1**	**95**	96.9
PRI [11]	84.9	93.5	96.1
LA-transformer [64]	86.7	*96.4*	**97.4**
Ours	**90.9**	**96.4**	**97.6**

The best and second-best results are in bold and italics, respectively.

**Table 2:** The proposed method is compared with the current state-of-the-art methods on the dataset CAVIAR.

Methods	CAVIAR		
	Rank-1	Rank-5	Rank-10
SING [12]	33.5	72.7	89
SPreID [60]	36.2	71.9	88.7
CamStyle [61]	32.1	72.3	85.9
CAD-net [62]	42.8	76.2	91.5
FFSR + RIFE [39]	36.4	72	—
CRGAN [63]	42.8	76.2	91.5
INTACT [22]	**44**	**81.8**	**93.9**
PRI [11]	43.2	78.5	91.9
LA-transformer [64]	42.1	80.7	92.4
Ours	**47.9**	**84.6**	**96.2**

The best and second-best results are in bold and italics, respectively.

**Table 3:** The proposed method is compared with the current state-of-the-art methods on the dataset MLR-CUHK03.

Methods	MLR-CUHK03		
	Rank-1	Rank-5	Rank-10
SING [12]	67.7	90.7	94.7
SPreID [60]	76.5	92.5	98.3
CamStyle [61]	69.1	89.6	93.9
CAD-net [62]	82.1	**97.4**	**98.8**
FFSR + RIFE [39]	73.3	92.6	—
INTACT [22]	**86.4**	**97.4**	**98.5**
PRI [11]	85.2	*97.5*	**98.8**
LA-transformer [64]	**86.3**	97.1	**98.6**
Ours	**91.8**	**97.5**	**99.2**

The best and second-best results are in bold and italics, respectively.

**Table 4:** Performance of different feature extractors on MLR-Market1501.

Structure	Weight learning	Rank-1	Rank-5
ResNet101	—	76.9	82.4
Two ResNet101	—	80.4	90.9
Two ResNet101	√	86.6	95.7
SR-DSFF (ours)	√	89.2	95.9

**Table 5:** The influence of different loss functions on recognition accuracy.

Loss functions	Rank-1	Rank-5	Dataset
Circle loss	88.4	95.7	MLR-Market1501
Triplet loss	88.7	94.9	MLR-Market1501
Sphere loss	89.3	96.1	MLR-Market1501
Ours	90.9	96.4	MLR-Market1501

**Table 6:** Performance of different feature extractors on MLR-Market1501.

Models	DS	Weight	Rank-1	Rank-5
CycleGAN [65]	—	—	62.6	76.2
SING [12]	—	—	74.4	87.8
CSR-GAN [66]	—	√	74.3	87.7
FFSR + RIFE [39]	√	√	66.9	84.7
CAD-NET [21]	—	—	83.7	92.7
SR-DSFF (ours)	√	—	86.1	92.6
SR-DSFF (ours)	√	√	90.3	96.4

“DS” represents whether dual-stream feature fusion is performed and “Weight” indicates whether weighting loss was added during feature extraction.

## Data Availability

The datasets used and analyzed during the current study available from the corresponding author on reasonable request.
